# Splenic Injury After Colonoscopy in a 55-Year-Old Female Patient

This article has been retracted.

**DOI:** 10.7759/cureus.35239

**Published:** 2023-02-20

**Authors:** Ilias Galanis, Magdalini Simou

**Affiliations:** 1 Second Department of Surgery, Evangelismos General Hospital, Athens, GRC

**Keywords:** post-colonoscopy injury, spleen hemorrhage, splenic trauma, splenectomy, colonoscopy complications

## Abstract

Colonoscopy is, in general, a relatively safe procedure with a low complication rate. Splenic injury related to this procedure is very rare, ranging from one in 100,000 to one in 6,387 colonoscopies, but a possibly lethal complication. For its diagnosis, a high degree of clinical suspicion is needed as many physicians are not aware of its existence. Clinical symptoms and signs are observed 1-10 days after the procedure. The imaging modality of choice is contrast-enhanced computed tomography (CECT). However, contrast-enhanced ultrasound (CEUS) may also be used to detect abdominal fluid and the injured area of the spleen. We present a case of a 55-year-old female with splenic rupture after a colonoscopy, diagnosed with CEUS and CECT. Splenectomy was performed, and the patient’s recovery was uneventful.

## Introduction

Colonoscopy is widely used in the last decades. Although a relatively safe procedure, it has its share of complications [1]. Splenic rupture constitutes a very rare but potentially life-threatening complication. Splenocolic adhesions, splenomegaly, anticoagulation therapy, and difficulty in performing the examination may be related [2]. Various pathogenetic mechanisms have been suggested, including direct trauma on the spleen and rupture of the splenic capsule due to traction of the splenocolic ligament or adhesions. Clinically, the patient presents with left upper abdominal quadrant pain, possibly radiating to the left shoulder, and peritoneal signs. Since colonoscopy is often performed with patient sedation, symptoms may be overlooked. Hypotension and decreased hemoglobin count may also be suggestive signs of splenic injury during colonoscopy [3]. Herein, we present the case of a 55-year-old female who presented with splenic rupture after an elective colonoscopy that had been performed five days earlier.

## Case presentation

A 55-year-old female presented to the emergency department complaining of left flank pain, fever, and malaise a few hours after a routine screening colonoscopy, which had been performed five days earlier without any significant findings. During this period of time, the pain had never subsided completely. On the contrary, it got worse during the last few hours. She was otherwise fit and well, with a past medical history of lumpectomy plus radiation therapy eight years ago for in situ ductal carcinoma of the breast and local resection and skin graft placement for squamous cell carcinoma of the scalp 10 years ago. She had no abdominal surgery, comorbidity, chronic home medication, or recent trauma. On admission, her blood pressure was 115/80 mmHg, her heart rate was 100 beats/minute, and she was hemodynamically stable. Mild tenderness and guarding especially over the left upper quadrant, without signs of peritonitis, were presented during physical examination. Initial workup revealed a hemoglobin concentration of 12.4 mg/dl and lactic acid level of 0.6 mmol/L.

Emergency ultrasound (US) revealed perisplenic fluid collection containing internal septations and debris, a finding suggestive of a non-acute hemorrhagic collection (Figure 1). A US contrast agent was injected intravenously, and contrast-enhanced US (CEUS) better outlined the collection, revealing its exact borders, while a filling defect in the lower part of the spleen, consistent with a splenic laceration, was observed (Figure 2).

**Figure 1:** US revealed perisplenic fluid collection containing internal septations and debris US: ultrasound

**Figure 2:** A filling defect in the lower part of the spleen, consistent with a splenic laceration

Computed tomography (CT) confirmed perisplenic hemorrhage and better imaged the patient’s splenic rupture. The patient was resuscitated with intravenous (IV) crystalloids and finally underwent exploratory laparotomy via a midline incision, which revealed hemoperitoneum, with 200-300 ml of bloody ascites. The splenic capsule was found to be detached from the splenic body at the inferior border, and there was a subcapsular hematoma at the anterior surface of the spleen (Figure 3).

**Figure 3:** Surgical specimen of the spleen

No colon perforation was found. An emergency splenectomy was performed, while a small splenunculus, which was found near the tail of the pancreas, was removed as well. The surgery lasted a total of one hour and a half with minimal blood loss.

Surgical pathology examination showed traumatic rupture of the spleen with no underlying splenic pathology and coexistence of a small splenunculus.

The patient’s recovery was uneventful, and she was discharged six days after the operation with guidelines for postsplenectomy vaccinations (pneumococcal, meningococcal, and *Haemophilus influenzae *type b {Hib} vaccinations). Her clinical condition nine months later was good.

## Discussion

Colonoscopy is a widely used screening method for colorectal cancer, for the diagnosis of large bowel pathology, and for therapeutic procedures [4]. It is a relatively safe method, both with and without sedation, and well tolerated by the patients [1]. Its complication rate is low, covering various entities. Mild complications include abdominal pain or distension, flatulence, nausea, and intestinal bleeding with no hemodynamic consequences [4]. The most common serious complications include hemorrhage (1%-2%) and perforation of the gastrointestinal tract (0.1%-0.2%) [1,5]. The latter is more frequently observed when polypectomy is performed [3,6] but usually does not require medical assistance [4].

Hemorrhage and perforation are responsible for the majority of the mortality rate of colonoscopy, especially when severe comorbidities are present [4], which, in any case, is low (0.006%-0.5% [7-9]). More infrequent complications include pneumothorax, pneumomediastinum, retroperitoneal emphysema, volvulus, hernia, incarceration, retroperitoneal abscess, vasovagal reaction, bronchospasm, endocarditis, and bacteremia [1]. The use of medication, condition of equipment, examination environment, endoscopist’s experience, intestinal preparation, mesentery or extracolic organ lesions, cardiovascular complications, and infection are also factors related to the rate of complications observed [4].

Iatrogenic splenic trauma related to colonoscopy is a dangerous and potentially lethal but rare complication, with an incidence of 0.004% [3]. It is more common when the patient has splenocolic adhesions due to previous surgery, pancreatitis, inflammatory bowel disease, and splenomegaly or has received oral anticoagulation treatment. Difficulty in performing the examination and techniques that lead to the torsion of the splenocolic ligament is also responsible for this complication [2]. In medical literature, the first case of colonoscopy-induced splenic injury was reported by Wherry and Zehner in 1974 [10]. Although more cases have been reported since [1,5,11-15], it is still a rare entity.

The exact pathogenesis of splenic trauma due to colonoscopy is not clear. Three different mechanisms have been suggested: a) direct injury on the spleen by the endoscope’s course through the splenic flexure, possibly with the addition of biopsy in the splenic flexure [1,2,11]; b) rupture of the splenic capsule caused by the traction of the splenocolic ligament; and c) rupture of the splenic capsule caused by the traction of adhesions (secondary to previous surgery, inflammation, or infection) between the spleen and the large bowel [1-3,11]. Splenomegaly (especially when the size of the spleen is over 15 cm) or underlying splenic disease has been suggested as factors increasing the incidence of splenic injury [16], as well as the distension of the large bowel by insufflated air [17].

A high degree of suspicion is needed for the diagnosis, as many doctors are not aware of this potential complication of colonoscopy, which may be fatal. Therefore, although rare, it needs to be considered when these symptoms arise after a colonoscopy with no evidence of colon perforation. The fact that colonoscopy is often performed with patient sedation, in order to decrease discomfort, results in diminished comprehension of pain and other signs of splenic trauma [3]. Symptoms and signs usually develop 24 hours after colonoscopy but may often occur up to 10 days later. In our patient, the symptoms developed immediately after the colonoscopy and lasted for five days where it worsened, and as a result, she presented to our hospital. Possibly, peristaltic or bowel movements may have played a role. Symptoms usually include left upper abdominal quadrant pain, possibly radiating to the left shoulder, accompanied by peritoneal signs [3]. Hypotension and decreased hemoglobin count without rectal bleeding after the procedure are also observed [3].

The imaging modality of choice for trauma of the spleen, as well as the liver and kidneys, is contrast-enhanced CT (CECT) [1,2,11,18]. The addition of intravenous contrast agent is very important, as non-enhanced CT may raise the suspicion of intra-abdominal hemorrhage but may fail to detect the injured areas, and both non-contrast CT and CECT need to be ideally performed [19]. CECT is excellent for detecting laceration and subcapsular hematoma, as well as for differentiating them from perisplenic clot and hemoperitoneum and calculating the extent of splenic injury [17,20]. Our patient had a grade 3 splenic injury (subcapsular hematoma > 50% of the surface area, ruptured subcapsular or intraparenchymal hematoma ≥ 5 cm, and parenchymal laceration > 3 cm in depth), while a grade 1 injury (subcapsular hematoma < 10% of the surface area, parenchymal laceration < 1 cm in depth, and capsular tear), according to the American Association for the Surgery of Trauma (AAST) grading scale for splenic lacerations, is the most common after colonoscopy. Grade 5 injury, which is the most severe, refers to any injury in the presence of splenic vascular damage with active bleeding extending beyond the spleen into the peritoneum. In stable patients, CECT is useful for deciding operative or nonoperative treatment of the patient [2,11].

In unstable patients, abdominal ultrasound (US) can quickly and reliably detect free abdominal fluid [2]. In US, the same principle of contrast agent addition as in CT may be applied: US without contrast injection is very sensitive in detecting intra-abdominal fluid, but the injured areas of the organs can be easily overlooked [18]. Contrast-enhanced US (CEUS) has proved to be a useful alternative to CECT for imaging solid abdominal organ trauma [18]. It is easy and fast to perform by the patient’s bedside, with no radiation exposure for the patient. In addition, US contrast agents are not excreted by the kidneys; therefore, they can be administered safely to patients with renal failure, while the anaphylactoid reaction rate is lower compared to CT agents [18]. As a result, CEUS should be initially performed, when available, in patients with suspicion of abdominal solid organ injuries [5]. In our case, CEUS was not performed from the beginning as the contrast agent was not available and should be brought from another hospital.

Therapeutic choices depend on the degree of splenic injury according to the American Association for the Surgery of Trauma (AAST) grading scale for splenic lacerations (Table 1) and the condition of the specific patient. Stable patients with ongoing hemorrhage are treated by splenectomy or selective embolization of the splenic artery, when available. If the patient is in hypovolemic shock, stabilization should be established before surgery. If the patient is a nonresponder to conservative treatment, surgical intervention should not be delayed. Spleen-preserving surgery by wrapping the organ in a Vicryl® net can be an alternative. Diagnostic laparoscopy can be helpful in assessing the extent of the injury in hemodynamically stable patients and preserving the spleen. In addition, in the setting of ongoing hemorrhage, selective embolization of the splenic artery, with coils or particles or a combination of both, may also be performed. This is a good option for unstable patients whose perioperative risk is high [3]. If the degree of subcapsular hemorrhage is low (AAST grade 1), the patient can be treated conservatively, but this is not the case for unstable patients and those with splenomegaly and other preexisting pathological conditions or upon hemoperitoneum [11].

**Table 1:** AAST spleen injury scale AAST: American Association for the Surgery of Trauma

Grade	Splenic injury
Grade 1	Subcapsular hematoma < 10% surface area, parenchymal laceration < 1 cm depth, and capsular tear
Grade 2	Hematoma: subcapsular, 10%-50% surface area; subcapsular hematoma, 10%-50% surface area; intraparenchymal hematoma, <5 cm; and parenchymal laceration, 1-3 cm
Grade 3	Subcapsular hematoma > 50% surface area, ruptured subcapsular or intraparenchymal hematoma ≥ 5 cm, and parenchymal laceration > 3 cm depth
Grade 4	Any injury in the presence of a splenic vascular injury or active bleeding confined within the splenic capsule, parenchymal laceration involving segmental or hilar vessels producing >25%, and devascularization
Grade 5	Any injury in the presence of splenic vascular injury with active bleeding extending beyond the spleen into the peritoneum

In our patient, baseline unenhanced US revealed perisplenic fluid collection with internal septa and debris, due to the fact that the hemorrhagic collection was not recent, since five days had passed since the colonoscopy. On CEUS, the hemorrhagic collection was better outlined, and a splenic laceration was seen. Subsequent CECT confirmed perisplenic hemorrhage and imaged the patient’s splenic rupture.

The patient was operated, and splenectomy was performed due to the fact that this grade of spleen injury could not be managed with conservative technique. The spleen, with the addition of a small splenunculus, was removed. Pathology confirmed splenic rupture with normal texture of the intact splenic parenchyma and no underlying pathology.

## Conclusions

Colonoscopy-related splenic rupture is a rare but dangerous complication. Physicians should be aware of its existence. Patients should be informed about possible colonoscopy complications. In case the patients complain of persistent abdominal pain after the procedure, they should be monitored and examined for potential splenic injury. The imaging modality of choice is CECT, while CEUS can be the initial examination.
